The article "Current Applications of Fecal Microbiota Transplantation in Functional Constipation" was published in 2022. Journal: Evid Based Complement Alternat Med.

# Current Applications of Fecal Microbiota Transplantation in Functional Constipation

**DOI:** 10.1155/2022/7931730

**Published:** 2022-07-13

**Authors:** Qi-Hong Liu, Xiao Ke, Cenxin Xiao

**Affiliations:** ^1^The Second People's Hospital Affiliated to Fujian University of Chinese Medicine, Fuzhou 350003, China; ^2^Fujian Clinical Medical Research Centre of Chinese Medicine for Spleen and Stomach, Fuzhou 350003, China

## Abstract

Functional constipation (FC) is a common condition that would be hard to treat in clinical practice with a prevalence incidence in the population. Pharmacotherapy is a common treatment modality. However, clinical effects are limited and patients continue to suffer from it. In recent years, with the gradual increase in research on gut microbiota, it is understood that dysbiosis of the gut microbiota is importantly associated with the development of constipation. Recent studies have shown that fecal microbiota transplantation (FMT) is an effective method for restoring gut microbiota, as well as being efficacious in the treatment of FC. This mini review explains the characteristics of gut microbiota in FC patients, the mechanism of action of FMT, treatment modalities, current efficacy, and related problems. The purpose is to provide research directions and references for the future applications of FMT in FC.

## 1. Introduction

Functional constipation (FC) is one of the more common diseases and is a form of chronic constipation. Patients may experience difficulty in defecation, a feeling of incomplete defecation, reduced frequency of defecation, and dry, hard stools, with the majority of elderly patients and women [1]. The exact pathogenesis of the disease is not yet clear, making it difficult to treat, and the recurrence of symptoms has a serious impact on the quality of human life. Patients often choose oral laxatives to treat constipation; although it can quickly relieve the symptoms of constipation, long-term use can easily lead to an imbalance of intestinal flora and even damage the function of intestinal nerves and smooth muscle, so that the sensitivity of the intestine is reduced, and the symptoms of constipation will be worse than before after stopping the drug. Therefore, it is essential to find a safe and effective measure to treat FC. In recent years, the contribution of microecological agents has led to a better understanding of FC and intestinal flora and the derivation of the emerging microecological therapy, fecal microbiota transplantation (FMT), by re-establishing the intrinsic microecological balance of the intestine [2]. FMT provides a new solution to address diseases in and out of the intestinal tract by rigorously screening the fecal sources of healthy donors and transplanting functional flora from healthy human feces through to the patient's intestine, thereby reregulating the distribution pattern of flora in the intestinal lumen and thus restoring the intestinal microecosystem to normal. FMT has been found to play a role in the treatment of FC in recent studies, but there is currently a large variation in reporting among research centers, the total number of cases studied is small, and the technical criteria used vary somewhat [3]. Therefore, in this paper, we review the characteristics of the intestinal flora of FC patients, the mechanism of action of FMT, treatment modalities, and the current status of efficacy, taking into account the literature reports related to FMT in the treatment of FC, in order to provide a reference for the standardized clinical use of FMT in the treatment of FC.

The article "Current Applications of Fecal Microbiota Transplantation in Functional Constipation" was published in 2022. Journal: Evid Based Complement Alternat Med.

### 1.1. Characteristics of Gut Microbiota in Patients with FC

Compared to healthy individuals, FC patients showed significant differences in the number and structural composition of intestinal flora. The identification of the changing characteristics of the gut microorganisms in FC patients is a prerequisite for the precise treatment of FMT. Zoppi et al. [4] performed fecal bacterial cultures on FC children and found a significant increase in *Bifidobacterium*. However, bacterial culture (Khalif et al. [5]) and Rt-PCR detection (Kim et al. [6]) of feces from adult FC patients showed a significant reduction in *Bifidobacterium* abundance. An analysis of the intestinal flora of elderly FC patients pointed to a significant increase in *Bifidobacterium* [7]. In view of the abovementioned contradictions in the research results of *bifidobacteria*, on the one hand, it is emphasized that although there is no doubt that *bifidobacteria* are currently used as probiotics for the human body, they can regulate intestinal flora, inhibit inflammation, and regulate metabolic pathways through three mechanisms to control the occurrence of FC [8]. However, it should also be recognized that FC patients of different ages may have unique intestinal flora characteristics, so the application of FMT should pay attention to the classification of age groups. On the other hand, it also revealed that early studies mostly used microscopy directly to assess standard microbial cultures by selective cultures, which lacked reproducibility and could not detect live and dead microorganisms in fecal samples, and there were errors in the determination of intestinal flora; meanwhile, traditional molecular biology assays reduced the objectivity of results due to their low throughput. Therefore, with the development of modern macro genomics, the determination of intestinal microbiota is now dominated by 16SrRNA.

The article "Current Applications of Fecal Microbiota Transplantation in Functional Constipation" was published in 2022. Journal: Evid Based Complement Alternat Med.

Zhu et al. [9] first used 16SrRNA to study the intestinal flora of FC children and found a significant decrease in Prevotella and an increasing trend in the thick-walled phylum. It has been demonstrated that Prevotella plays a key role in the development and treatment of constipation, so a decrease in its abundance is likely to be associated with FC [10]. Mancabelli et al. [11] showed that the intestinal flora of FC patients had a significant decrease in *Bacillus spp*, *Rhodobacter spp,* and *Faecaloccus spp*. The above studies mainly inferred the intestinal microbiota composition through the fecal microflora study, which lacked attention to the intestinal mucosal microflora. Therefore, Parthasarathy et al. [12] collected mucosal and fecal microbiota samples from the sigmoid colon of female patients with chronic constipation, evaluated them by 16SrRNA gene sequencing, and found that *Bacteroidetes* were more abundant in the colonic mucosal microbiota of patients with constipation. It is also noted that the intestinal flora of constipated patients has a unique microbiota on both the colonic mucosa and the feces, where the colonic mucosa is not affected by diet and colonic transport, while the fecal bacteria are disturbed by colonic transport, but are not associated with constipation. Thus, the intestinal flora of FC patients has a unique microbiota on both the colonic mucosa and the feces, where the colonic mucosa is not affected by diet and colonic transport, while the fecal bacteria are disturbed by colonic transport, but not by constipation. This may be one of the reasons for the same study methods with contradictory results.

In addition, environmental factors, dietary habits, medication, and intestinal dynamics may be potential factors affecting the composition of the intestinal flora of FC patients [13] Fecal characteristics also affect the distribution of intestinal flora, and studies have shown that species richness is positively correlated with fecal water content and negatively correlated with fecal hardness [14]. However, the lack of uniformity in the flora species derived from current trial findings reduces comparability, and the current 16SrRNA assay can only address bacterial taxonomy at the genus level and above. Therefore, screening for more similar test groups and developing more refined study criteria are necessary to improve the accuracy of gut flora results in FC patients and provide more targeted treatment for the use of FMT.

### 1.2. Mechanism of FMT for FC

Microbial communities are found on the surface of the human body and in the external lumen, with the highest density found in the distal intestine, where they far exceed the total number of cells in the body. In fact, the distal gut flora is thought to have a variety of physiological functions, including energy metabolism, development of the immune system, and regulation of various body organs [15]. Recent studies have shown that the structure of intestinal flora is abnormal in patients with constipation, with a significant increase in the number of potentially pathogenic bacteria (aerobic bacteria, Escherichia coli, and fungi) in the stool on the one hand and a significant decrease in the number of dominant flora (anaerobic bacteria, bifidobacteria, and anaphylactic bacteria) on the other hand [16]. Intestinal flora disorders can be involved in the development and progression of FC through various pathways including the nervous system and intestinal flora metabolites. 5-Hydroxytryptamine is a neurotransmitter in the brain-gut-bacteria axis, and Bifidobacterium bifidum induces an increase in 5-hydroxytryptamine secretion. The metabolites of intestinal flora speed up colonic transmission by promoting the secretion of 5-hydroxytryptamine; FC patients with reduced dominant flora cannot effectively promote the secretion of 5-hydroxytryptamine, thus causing constipation [17]. FMT transplants healthy human intestinal flora into the patient's intestine through a suitable pathway to rebuild the microecology of the intestinal microbiota, normalize the composition and function of the intestinal microbiota, regulate intestinal mucosal immunity and intestinal barrier function, and restore intestinal dynamics, thereby alleviating the symptoms associated with constipation [18]. In addition, FMT administration via colonoscopy rapidly induced microbiological normalization of the community structure, and its intestinal flora 24 h after administration was very similar to the composition of the donor [19].

The article "Current Applications of Fecal Microbiota Transplantation in Functional Constipation" was published in 2022. Journal: Evid Based Complement Alternat Med.

## 2. Treatment of FMT

### 2.1. Source of Fecal Bacteria

The selection of fecal source is the result of bidirectional selection of donor and recipient, and standardized screening of donor fecal samples can guarantee the safety of recipient transplantation while clarifying the altered intestinal flora of the recipient can ensure the relevance of donor selection. First, the source of fecal bacteria is currently selected from family members, friends, or standardized fecal bacteria banks. For long-term fecal donors, it is clearly proposed that a new round of screening should be performed at 8–12 weeks and even emphasizes the importance of diet, exercise, and health management of donors during the transplantation cycle to reduce the disturbance of fecal samples by external uncertainties, which ensures the safety of the fecal source to a certain extent and reduces the potential factors affecting the composition of the flora [20]. Secondly, the storage of fecal sources has now formed a standardized process that requires the preparation to be completed within 6 h of donation and stored in a −80°C refrigerator for a storage period of no more than 6 months. Finally, the transplantation of the fecal source, whether it comes from the same donor, is unclear. The goals of FMT transplantation are to reduce the interference of different fecal sources with the outcome, to avoid recipient graft rejection, and to promote the reconstitution of the intestinal flora in FC patients. Thus, bidirectional matching for donor-acceptor can now be grouped into 2 models as follows: (1) One-to-one (one subject for one donor), although this model clarifies the correspondence, is there a rapid saturation of a certain flora in the recipient after multiple transplants, leaving other beneficial bacteria not yet at optimal the possibility of a stoppage in efficacy occurring because other beneficial bacteria have not yet reached optimal numbers. (2) One-to-many (one subject corresponds to multiple donors), with the possibility of rejection of colonization between beneficial bacteria and weakening of efficacy occurring when fecal sources from different donors are transplanted into the recipient's intestine. It follows that in multiple sessions of FMT transplantation, additional one-to-one fixed pairs or one-to-many random pairs can be added to narrow down the influencing factors that lead to diminished efficacy.

### 2.2. Fecal Bacteria Implantation Method

Fecal bacteria implantation is mainly given by 3 digestive tract modalities: upper, middle, and lower. In an analysis of the effectiveness of a trial of treating FC patients by different routes of administration (oral capsule, nasogastric tube, and colonoscopy), it was suggested that the differences between the groups were statistically significant [21]. However, there is insufficient evidence to confirm that one mode of delivery is the most appropriate, and there are two sides to any one delivery method. There are two sides to any method of administration. The upper gastrointestinal route is dominated by the nasogastric tube, the oral capsules as the dominant route, and the presence of which makes it difficult to ensure complete coverage of the fecal fluid in the entire intestinal tract, increasing the potential for small intestinal bacterial overgrowth. At the same time, the placement of the nasogastric tube can easily cause the subjects to have uncomfortable reactions such as vomiting, which is accompanied by an increased risk of aspiration. The use of oral capsules is now preferred because of their simplicity and convenience, which greatly avoids the discomfort of instrumental intrusion. However, due to the rigorous and costly preparation and storage process, the economics are challenging and PPI preparations are often required to reduce the concentration of gastric acid in order to avoid damage to the effectiveness and stability of the capsules. The lower gastrointestinal route is more commonly known as enema and colonoscopy. Enemas rely on the reverse flow of fecal fluid into the colon and are mostly confined to the splenic flexure of the colon and the following segments. Colonoscopy allows the fecal fluid to be distributed more evenly throughout the intestinal tract along with the peristaltic process, but because of the invasive nature of the procedure, there is a risk of intestinal perforation and, in some patients, transient diarrhea. In conclusion, the most appropriate regimen should be selected after an individual assessment of the patient's compliance and tolerability.

The article "Current Applications of Fecal Microbiota Transplantation in Functional Constipation" was published in 2022. Journal: Evid Based Complement Alternat Med.

## 3. Current Status of FMT Efficacy

### 3.1. Frequency of Transplantation

The frequency of FMT migration in FC patients has been studied in 2 ways in the majority of studies: (1) single course of transplantation: the main model is a course of treatment of 1 time/d for 3 d. Tian et al. [22] in the study of FMT-treated FC patients, with complete spontaneous defecation ≥ 3 times as the criterion for clinical remission rate, monitored changes at weeks 1, 2, and 4 during follow-up, reaching optimal values at week 4. Ge et al. [23] treated 21 patients with STC with FMT using the same judgment criteria, again reaching a maximum level at week 4, with a decline in efficacy at week 12 of follow-up. In order to track the long-term duration of FMT, Ding et al. extended the follow-up period to 24 weeks, and although the clinical remission rates at weeks 3–4, 9–12, and 21–24 were significantly better than before treatment, the efficiency rate gradually decreased from week 12 onwards, reaching a minimum at week 24. Therefore, FMT is effective in relieving the existing clinical symptoms of FC patients and has a positive impact on the recovery of bowel motility and defecation function. FMT is a remodeling process in which the hosts gut changes from colonization resistance to compatibility with the transplanted bacteria. When the transplanted bacteria and the host flora reach an optimal state of mutual integration, they re-establish a new intestinal flora equilibrium, restoring the number and composition of the intestinal flora to that of a healthy person, but with a tendency to decline again over time as the transplanted bacteria do not settle permanently in the host intestine. A single course of FMT treatment has better short-term than long-term efficacy, and 1 to 3 months appears to be the turning point in the persistence of FC patients. (2) Multiple transplants: one or more FMT per session, with a certain interval between sessions. Zhang et al. administered a total of 3 courses of FMT (1 time/d for 6 d, repeating a course after 1 and 3 months) to patients with FC, assuming complete spontaneous defecation ≥ 3 times as the criterion for clinical remission, with a decreasing trend in remission rates from week 4 onwards, again confirming that short-term efficacy (4 weeks) was superior to long-term efficacy (1 year) [24]. In addition, in a total of 34 patients with FC, the Wexner constipation score of < 8 was used as the criterion for a cure during 3 courses of FMT (1 course each, 3 weeks apart), and the results of the 5 follow-up visits at the end of each course and the second and third months after the last treatment were compared, with the patients' symptoms improving without any significant rebound and the overall clinical cure rate reaching 73.5% [25]. Multiple FMT interventions in patients with FC appear to facilitate the consolidation of overall efficacy, enhance the ability of beneficial bacteria to reside in the gut, slow their decay, and maintain the gradual formation of a state of equilibrium in the gut in a new environment, a pattern of treatment that somewhat diminishes the loss of efficacy. However, the timing of multiple FMT treatments is still inconclusive, and further research is needed to maximize the benefits of FMT interventions to promote the long-lasting survival of beneficial bacteria in the body's gut.

The article "Current Applications of Fecal Microbiota Transplantation in Functional Constipation" was published in 2022. Journal: Evid Based Complement Alternat Med.

### 3.2. Duration of Transplantation

In addition to the possible impact of differences in transplant frequency on clinical efficacy, the duration of FMT may be related to the following factors [26]: (1) The mechanism of short-term efficacy is unknown: the construction of foreign beneficial bacteria transplanted into the organism is the final outcome of the mutual competition between colonization and resistance, and there is a lack of research on the mechanism of superior short-term efficacy. (2) Saturation and colonization rejection of fecal bacteria: at this stage of multiple courses of transplantation, the changes in the intestinal flora of FC patients after each course of treatment have not been focused on for the time being, considering the differences in colonization and recovery of the intestinal flora of different individuals, and whether there is a difference in the time frame for saturation of the transplanted flora between individuals without changing the fecal source. The outcome revealed by the use of a different fecal source for each session is an open question as to whether the later transplanted community forms a colonization rejection contest against the previous resident community. (3) Antibiotic use: FC patients after FMT treatment cannot avoid the situation that none of them will use antibiotics for a short period of time, and the effect of the antimicrobial drug concentration in the colon on the colonization effect of transplanted bacteria is unclear on the basis of rational use, and intestinal flora disorders may occur again. (4) Others: China's first FMT methodological consensus opinion points out that age, disease duration, diseases, or drugs that significantly affect the intestinal flora may interfere with the efficacy of FMT. In addition, whether the types of FC, transplantation method, and selection of fecal source for multiple treatments have statistical differences in the efficacy and the effect on the homeostatic construction of the transplanted flora are to be evaluated in more depth, so as to find the optimal treatment for FMT and reduce the adverse effects and economic burden on patients.

### 3.3. Combination Therapy

The efficacy of FMT alone in treating FC has been demonstrated [27]. Based on the current status of research, the FMT combination can be summarized into 2 forms. (1) Combination of western drugs: osmotic laxatives are classically used in FC, and the combination with FMT produces a more significant synergistic effect. Liu et al. [28] used FMT in combination with polyethylene glycol electrolyte dispersion, and the experimental group showed a 30% improvement in symptoms compared to the control group. In addition, Ge et al. [23] formulated pectin on the basis of FMT and the results were also better than those of the FMT group. The combination of FMT with western drugs consolidates the colonization of transplanted bacteria in the host intestine and reduces the loss of transplanted bacteria, thus demonstrating an increase and persistence of efficacy. (2) United Herbal Medicine: Zhang et al. [29] treated FC with FMT combined with fluid-enhancing Cheng qi Tang, which was superior to the FMT group in terms of gastrointestinal electrical amplitude and clinical symptoms. A study combining Liu Wei Neng Xiao Capsules for the treatment of FC patients with Spleen Qi weakness suggested a higher clinical improvement rate than the FMT group. With a little laxative, it may be possible to obtain better benefits. There is a lack of research on the mechanism of FMT combined with Chinese medicine treatment. The current research focus should be on the long-term efficacy of FMT while exploring the clinical value of combination therapy [30].

The article "Current Applications of Fecal Microbiota Transplantation in Functional Constipation" was published in 2022. Journal: Evid Based Complement Alternat Med.

## 4. Current Problems

At present, the standardization of FMT is gradually receiving attention, and the consensus opinion of experts in China has clearly proposed that the donor screening standards and the FMT operating procedures for fecal liquid preparation. FMT has the characteristics of foreign organ implantation at some level, which involves ethical issues, how to select the appropriate flora for the recipient's intestinal microenvironment, how to match the transplantation relationship between the donor and recipient, how to avoid the rejection reaction after transplantation, and how to construct a follow-up model for monitoring. Second, the advantages and disadvantages of transplantation routes, the efficacy of FMT, and the advantages of combination drugs have received attention, but the lack of large sample size and prospective clinical studies to support the optimal route, optimal transplantation frequency, and optimal combination drugs, as well as the lack of consensus on the best guidelines to guide them, coupled with many external influencing factors, individual differences, and other uncontrollable conditions, have once again made the clinical work more challenging. Identifying the characteristic intestinal flora changes of FC patients and exploring the best means of implementing FMT will not only improve the clinical symptoms of patients but also standardize the treatment of FC by FMT. In addition, it is important to enhance the public awareness of FMT and eliminate patients' psychological concerns about the operation in order to enhance the clinical use of FMT and lay a solid foundation for the safety, individualization, and long-term effectiveness of FMT for FC.
